# Sulforaphane Ameliorates Limb Ischemia/Reperfusion-Induced Muscular Injury in Mice by Inhibiting Pyroptosis and Autophagy via the Nrf2-ARE Pathway

This article has been retracted.

**DOI:** 10.1155/2022/4653864

**Published:** 2022-05-11

**Authors:** Huanhuan Sun, Jueqiong Wang, Wei Bi, Feng Zhang, Kui Chi, Long Shi, Tao Yuan, Kai Ma, Xiang Gao

**Affiliations:** ^1^Department of Vascular Surgery, The Second Hospital of Hebei Medical University, Shijiazhuang 050000, Hebei, China; ^2^Department of Neurology, Neurological Laboratory of Hebei Province, The Second Hospital of Hebei Medical University, Shijiazhuang 050000, Hebei, China

## Abstract

**Background:**

Limb ischemia/reperfusion (I/R) injury, as a life-threatening syndrome, is commonly caused by skeletal muscle damage resulting from oxidative stress. Additionally, inflammation-induced pyroptosis and dysregulated autophagy are vital factors contributing to the aggravation of I/R injury. Of note, sulforaphane (SFN) is a natural antioxidant, but whether it worked in limb I/R injury and the possible mechanism behind its protection for skeletal muscle has not been clearly established.

**Methods:**

Effects of SFN on limb I/R-injured skeletal muscle were assessed by HE staining, followed by assessment of wet weight/dry weight (W/D) ratio of muscle tissues. Next, ELISA and biochemical tests were used to measure the inflammatory cytokine production and oxidative stress. Immunofluorescent analysis and Western blot were adopted to examine the level of pyroptosis- and autophagy-related proteins *in vivo*. Moreover, protein levels of Nrf2-ARE pathway-related factors were also examined using Western blot.

**Results:**

SFN treatment could protect skeletal muscle against limb I/R injury, as evidenced by diminished inflammation, pyroptosis, autophagy, and oxidative stress in skeletal muscles of mice. Further mechanistic exploration confirmed that antioxidative protection of SFN was associated with the Nrf2-ARE pathway activation.

**Conclusions:**

SFN activates the Nrf2-ARE pathway, and thereby inhibits pyroptosis and autophagy and provides a novel therapeutic strategy for the limb I/R-induced muscle tissue damage.

## 1. Introduction

Limb ischemia/reperfusion (I/R) injury represents a life-threatening disease owing to arterial embolism, primary thrombosis, artery transplantation, limb or flap reattachment, trauma, and abdominal compartment syndrome [1]. Patients with mild I/R injury may suffer from fibrosis, and permanent damage and necrosis in the skeletal muscle; in severe cases, patients may develop syndromes of multiple organ dysfunction [2].

Recent studies indicate that pyroptosis may be responsible for the pathogenesis of I/R injury [3–5]. Pyroptosis induced by I/R is mediated by activation of NLRP3 inflammasome, which is a multiprotein complex comprising of ASC, NLRP3, and pro-caspase-1. It can be activated in the presence of danger signals and trigger the release of IL-1*β* and IL-18 via activation of pro-caspase-1 [6–8]. Excessive inflammatory responses play key roles in the pathogenesis of I/R [9]. Therefore, targeting pyroptosis and inflammation could be essential therapeutic strategies for limb I/R injury treatment.

Autophagy, a highly-conserved system, is essential for homeostasis and cellular integrity maintenance in eukaryotic organisms. It can be induced by various intra- and extracellular injuries, including hypoxia, starvation, inflammation, and endoplasmic-reticulum stress-caused injuries. Notably, autophagy closely links to the pathogenesis of I/R injury [10, 11]. Autophagy captures the cellular organelles and damaged proteins in autophagosomes [12]. The production of autophagosomes is dependent on activation of several genes, such as LC3, autophagy-related genes (Atgs), and beclin-1 genes [13]. Therefore, we infer that modulating autophagy may be an effective strategy to treat I/R injury.

Overproduction of ROS occurs in I/R-injured organs and oxidative stress may associate with development of skeletal muscle I/R injury [14, 15]. Antioxidant enzymes, including SOD, GPx, NADPH, NQO1, and HO-1, can protect cells against oxidative stress. Nrf2, a member of the NFE2 family of transcription factors, represents a major regulator of the abovementioned cytoprotective enzymes [16–20]. Moreover, recent studies have also reported that Nrf2 pathway could modulate pyroptosis by inhibit NLRP3 inflammasome activation. ROS not only acts as messengers in cell survival, death, and immunity pathways [21] but also activates autophagy [22–25]. Nrf2 pathway can also modulate autophagy. These studies suggest crosstalks among oxidative stress, pyroptosis, and autophagy. Therefore, exogenous antioxidants represent a useful adjunctive option or a beneficial therapeutic strategy for limb I/R injury treatment.

A natural compound, sulforaphane (SFN), predominantly existing in cruciferous vegetables [26], is essential for cellular redox balance maintenance [27]. SFN has been earlier used as an effective antioxidant in the investigation into various diseases, including I/R injury. In addition, SFN can suppress multiple inflammasomes in immune cells [28]. SFN has the potency to protect pancreatin acinar cell injury owing to its regulation on NLRP3 inflammatory pathway and Nrf2-mediated oxidative stress; meanwhile, it can prevent obesity-driven damage to the reproductive system of male mice by modulating autophagy and oxidative stress [29, 30]. Therefore, we inferred that SFN, serving as an antioxidant, may alleviate limb I/R injury-induced muscular injury by modulating pyroptosis and autophagy via the Nrf2-ARE pathway. The aim of this study is to elucidate the protective effect of SFN on skeletal muscles from limb I/R injury and to determine the underlying mechanism associated with such beneficial effects.

## 2. Methods and Materials

### 2.1. Animals and Ethics Statement

In this study, male C67/BL6 mice (8–10 weeks, 23–25 g; obtained from the SPF (Beijing) Biotechnology Co., Ltd) were housed with sufficient food and water. All experiments were approved by Ethics committee of Hebei Medical University and conducted based on the Guide for the Care and Use of Laboratory Animals (National Institutes of Health).

### 2.2. Mouse Models of Femoral Artery I/R

Femoral artery and vein of mice were exposed. The supply of blood was blocked using an atraumatic microvascular clamp, and a band was fitted around the left thigh to induce ischemia for 1.5 h. Next, the clamp and the band were removed to induce reperfusion for 72 h before sampling.

### 2.3. Experimental Protocols

All mice were randomly grouped into sham, I/R and I/R + SFN (5 mg/kg; Shanghai Bide Pharmatech Ltd.) groups. The femoral arteries and veins of mice in sham group were only isolated for 1.5 h while those of mice in I/R group were blocked for 1.5 h. The two group of mice were intraperitoneally administered saline prior to reperfusion on the day of surgery, and the mice were intraperitoneally administered saline once on a daily basis for two additional days prior to sampling. In I/R + SFN group, mouse femoral artery and vein were blocked for 1.5 h. The mice were intraperitoneally administered saline through an injection containing 5 mg/kg SFN prior to reperfusion on the operation day and the drug treatment was given once per day for two additional days prior to sampling.

### 2.4. Histological Examination

Following three days of drug treatment, the pretibial muscle tissues were carefully dissected and embedded in paraffin. Muscular sections (5 *μ*m) were stained with HE for assessing the general histology and inflammation. Regarding the histological assessment of limb muscular injury, three random fields were calculated for impairment. Healthy fibers were identified with possessing complete borders arrayed regularly with no holes, breaks, and edema. Meanwhile, injured fibers were accompanied by edema resulting in broken and fragmented fiber. The degree of inflammation was evaluated as previously described [9].

### 2.5. Wet Weight/Dry Weight (W/D) Ratio of Muscle Tissues

The pretibial muscle of the mice was weighed instantly once it was removed from the left hind limb (wet weight). The muscles were weighed once more after they were dehydrated (dry weight). The degree of edema in the muscle tissue was evaluated using the W/D ratio as follows: W/D ratio = (wet weight/dry weight) × 100% [9].

### 2.6. ELISA

ELISA kits (ELK1271, ELK2269, ELK1395, ELK1157, ELK Biotechnology, Wuhan, China) were adopted to determine the levels of IL-18, IL-1*β*, IL-6, and TNF-*α* in the homogenate of muscle tissues.

### 2.7. LDH, CK-MB, MDA, and SOD Measurement

The production of MDA was measured using a MDA detection kit (A003-1, Jiancheng Biotechnology, Nanjing, China). The activity of SOD (A001-3) and levels of LDH, and CK-MB in muscular homogenate were measured using commercial kits (A020-1, E006-1-1, Jiancheng Biotechnology).

### 2.8. Immunofluorescent Staining

Muscle tissue sections (5 *μ*m) were probed overnight at 4°C with antibodies to Beclin-1 (1 : 100, A7353, Abclonal), LC3 (1 : 200, 14600-1-Ap, Proteintech, China) and caspase-1 (1 : 100, DF6148, Affinity). The sections were re-probed with a secondary antibody for 50 min and stained with DAPI for 5 min. After mounting, immunofluorescent signaling was observed with a fluorescence microscope to evaluate the extent of pyroptosis.

### 2.9. Western Blot

Muscle tissues were lysed with a RIPA buffer. The samples of protein were boiled with loading buffer before separation with SDS/PAGE, followed by transfer to a PVDF membrane. Primary antibodies used in this assay included caspase-1 (af5418, 1 : 500, Affbiotech), NLRP3 (^#^15101; 1 : 500, Cell Signaling Technology [CST], Danvers), ASC (bs-6741R; 1 : 500; Bioss Technology, Beijing, China), Belcin-1 (^#^3738; 1 : 1000, CST), LC3 (^#^4108; 1 : 1000, CST), p62 (ab109012; 1 : 10000; Abcam, UK), Nrf2 (ab137550 1 : 500; Abcam), HO-1 (^#^43966; 1 : 2000, CST), NQO1 (67240-1-Ig, 1 : 1000, Proteintech), and GAPDH (ab37168; 1 : 10000; Abcam). Following probing with the above antibodies, the membrane was re-probed with a secondary antibody (AS1107, 1 : 10000; ASPEN, Wuhan, China). ImageJ software was applied for quantitative analysis.

### 2.10. Statistical Analysis

Statistical analysis, by SPSS 19.0 software, include Bonferroni-corrected one-way ANOVA for multi-group numerical data difference, with the data summarized as mean ± SD. *p* < 0.05, *p* < 0.01 was statistically significant.

## 3. Results

### 3.1. SFN Alleviated I/R Injury-Induced Muscular Injury

H & E staining was used for evaluating muscle tissue injury. Healthy fibers were identified by the complete borders that were regularly arrayed with no holes, breaks, and edema. On the other hand, injured fibers were accompanied by edema and the fiber was broken and fragmented. Muscle fiber degeneration, sarcoplasm, dissolution, inflammatory cell infiltration, and myoedema were seen in the I/R group; however, such conditions were not visible in the sham group. SFN treatment alleviated the degree of inflammation of muscle tissues of I/R mice (Figure 1(a)). Consequently, SFN treatment in I/R mice alleviated the pathological scores in muscle tissues induced by the I/R injury (Figure 1(b)).

Furthermore, the W/D ratio of skeletal muscle tissues was determined to assess tissue edema in muscular injury. Resultantly, a higher W/D ratio was observed in I/R group versus sham group (Figure 1(c)). Moreover, the W/D ratio of skeletal muscle tissues in SFN group was lower than that in I/R group (Figure 1(c)).

### 3.2. SFN Ameliorated Inflammatory Response in Skeletal Muscle of Mice with Limb I/R Injury

Levels of IL-18, TNF-*α*, IL-1*β*, and IL-6 were remarkably higher in the I/R group versus the sham group. Evidently, SFN treatment in I/R mice alleviated the increments in these cytokine levels triggered by I/R injury. Moreover, the I/R group had higher levels of LDH and CK-MB than the sham group, indicating the incidence of neutrophil infiltration and inflammatory cytokine secretion following I/R. SFN treatment led to noticeably attenuated levels of LDH and CK-MB (Figure 2).

### 3.3. SFN Suppressed Limb I/R-Induced Pyroptosis in the Skeletal Muscle Tissues of Mice

Immunofluorescent analysis labelled caspase-1 was used to observe the level of pyroptosis in different groups of mice. High expression of caspase-1 was found in the I/R group while with SFN treatment, the increased expression of caspase-1 upon I/R injury was reduced (Figure 3(a)).

In addition, Western blot data presented augmented expression of pyroptosis-related proteins (NLRP3, ASC, and caspase-1) in I/R group while it was reduced following SFN treatment (Figures 3(b) and 3(c)).

### 3.4. SFN Downregulated Limb I/R-Induced Autophagy in the Skeletal Muscle Tissues of Mice

To investigate whether SFN treatment could influence autophagy in the muscle tissue of mice. Immunofluorescent analysis labelled autophagy markers Beclin-1 and LC3 was used to observe the level of autophagy. I/R injury increased level of autophagy, as shown by higher expression of LC3 and Beclin-1 in I/R group versus sham group. Moreover, SFN treatment lowered the expression of Beclin-1 and LC3 in the I/R mice (Figure 4(a) and 4(b)).

Western blot results showed higher Beclin-1 expression but lower p62 expression in I/R group relative to sham group, while there was lower Beclin-1 expression but higher p62 expression in the SFN group than in the I/R group. Additionally, I/R resulted in increased LC3II/LC3I ratio, which was rescued by SFN (Figures 4(c) and 4(d)).

### 3.5. SFN Alleviated Oxidative Stress in Skeletal Muscle Tissues of Mice with Limb I/R Injury

In comparison with the sham group, MDA production was higher in the I/R group. Additionally, versus I/R group, the lower production of MDA was detected in the SFN group (Figure 5(a)). Moreover, the lower SOD activity was considerably observed in I/R group versus sham group. Compared to the I/R group, the SOD activity was higher in SFN group (Figure 5(b)).

### 3.6. SFN Protected Skeletal Muscles of Mice against Limb I/R Injury by Activating Nrf2-Are Pathway

Nrf2/ARE and the associated antioxidant enzymes, including HO-1 and NQO1, function as key regulators for oxidative stress. We used Western blot to examine the effect of SFN treatment on the expression of Nrf2, HO-1, and NQO1 in the muscle tissue of mice. As illustrated in Figure 4, the expression of Nrf2, HO-1, and NQO1 was enhanced in the I/R group versus sham group. However, the expression of Nrf2, HO-1, and NQO1 was increased in the SFN group versus I/R group, suggesting that treatment with SFN, to some extent, activated Nrf2-ARE pathway in the muscle homogenate, to protect against limb I/R injury (Figure 6(a) and 6(b)).

## 4. Discussion

In the current research, we initially explored whether SFN could lessen limb I/R injury-induced level of inflammation and mitigate tissue edema in skeletal muscle. We also suggested that SFN could inhibit limb I/R injury-driven pyroptosis and autophagy. In addition, SFN was demonstrated to potentially protect the skeletal muscle against limb I/R injury by boosting Nrf2-ARE pathway to lessen oxidative stress, thereby suppressing pyroptosis and autophagy.

Skeletal muscle damage induced by limb I/R injury represents an essential clinical issue [1, 2, 14]. There have been different strategies to treat limb I/R injury until now, including physical and chemical treatments. Previous research has indicated that hypothermia, ischemic preconditioning and postconditioning, light-emitting diode therapy, and controlled reperfusion could alleviate I/R-induced limb skeletal damage [31–33]. Furthermore, a few medications, including curcumin, dexamethasone, simvastatin, silibinin, hydrogen-rich, cyclosporine A, and saline [34–36], have been powerful in reducing intense skeletal damage initiated by limb I/R injury. However, such methods are limited in instances of horrendous wounds where I/R injury cannot be anticipated, and early intercession is required. In specific cases, particularly in serious extremity injuries, surgeries are performed to save lives and prevent hemorrhage to protect the functionalities of fundamental organs. Saving the extremities may not be the essential concern. In addition, despite the fact that the procedures and medication treatment referenced above have been demonstrated to be successful in the research facility, none has been confirmed to be effective in clinical settings. In this manner, there is a pressing need to explore novel agents with multiple characteristics that can be applied to treat the I/R-induced damage of skeletal muscle.

SFN has demonstrated numerous favorable effects, including neuroprotection, anti-inflammatory, antioxidant, and anticancer. In this study, we initially examined the potential of SFN against limb I/R injury and underlie the mechanism.

Pyroptosis is a new form of inflammatory necrosis regulating cellular immune and inflammatory responses, which lead to cell perforation and further cell necrosis [37, 38]. Recent studies indicate that pyroptosis can be induced by the I/R injury, which is mediated by NLRP3 inflammasome activation, resulting in bioactive IL-1*β* and IL-18 release [6–8]. Therefore, we inferred that inhibiting pyroptosis may be an effective strategy to alleviate I/R injury. Several studies have clarified that inhibiting pyroptosis could alleviate tissue damage induced by I/R injury. Some drugs, like Metformin, can delay intestinal I/R injury and cell pyroptosis through the TXNIP-NLRP3-GSDMD pathway [39]. In addition, SFN could inhibit NLPR3 inflammasome to alleviate retinal and cerebral I/R injury [40, 41]. However, whether SFN could mitigate muscular injury induced by limb I/R injury remains elusive. In this study, we found that SFN treatment could inhibit pyroptosis-related protein expression which is observed augmented upon I/R injury. These results indicate that SFN may mitigate muscular injury driven by limb I/R injury through inhibiting pyroptosis.

Defective, dysregulated and excessive autophagy have been intensively associated with I/R injury pathogenesis. Autophagy activation occurs in varied target organ models of the I/R injury, such as cerebral I/R injury, myocardial I/R injury, and intestinal I/R injury [42–44]. However, whether autophagy exerts protective or destructive effects following I/R remains unknown. Moderate autophagy can remove damaged organelles, thus facilitating cell survival, but excessive autophagy potentially causes cell death. Based on these, autophagy activation degree and persistence may determine the opposing effect. The variation in results may also be attributed to difference of species and sources of cells or of animal diseases used. For instance, in the context of spinal cord I/R injury, the early (8 h after injury) activated autophagy can reduce the injury via apoptosis and inflammation inhibition; yet the later (72 h after injury) excessive autophagy exacerbates the injury by stimulating autophagic cell death [45]. In our study, following 72 h of drug treatment, the pretibial muscle tissues were carefully collected for experiments. We found I/R injury increased level of autophagy and SFN treatment inhibited autophagy, thus alleviating limb I/R injury in the later stage. These results indicate that SFN may be a promising strategy to mitigate limb I/R injury-induced muscular injury through inhibiting pyroptosis.

Oxidative stress has been implicated in skeletal muscle I/R injury development [14, 15]. NQO1, SOD, HO-1, and GPx are well-known antioxidant enzymes of the Nrf2/ARE pathway [46]. Activation of Nrf2/ARE and the downstream genes demonstrates the protective effects against organ damage upon I/R injury [16, 17]. However, the pathophysiological mechanism of varied conditions, severity, and progression correspond to different influence on the Nrf2 expression [18, 19]. In this study, Nrf2 expression was higher in SFN group than the untreated control, and SFN treatment induced Nrf2 activation. In addition, concerning Nrf2 activation, we observed increased HO-1, NQO1, and SOD1 expression in response to SFN treatment. These findings agree with a previous work that SFN induces anti-oxidant responses in experimental autoimmune encephalomyelitis [20]. More importantly, SFN weakens pancreatin acniar cell injury via regulation of Nrf2-mediated oxidative stress; it also retards obesity-induced damage in the male mouse reproductive system via oxidative stress and autophagy [29, 30]. These studies may indicate the crosstalk among pyroptosis, autophagy and oxidative stress. It can be concluded that SFN may alleviate limb I/R injury-induced muscular injury by modulating pyroptosis and autophagy via activating Nrf2-ARE pathway.

## 5. Conclusion

In summary, this study revealed the protective properties of SFN against skeletal muscle damage induced by limb I/R injury, which was associated with inhibition of pyroptosis, autophagy, and oxidative stress via the Nrf2-ARE pathway. These findings highlight the potential of SFN as an effective drug strategy in the treatment of limb I/R injury-induced muscular injury.

## Figures and Tables

**Figure 1:** (a) HE staining was used to observe degree of inflammation of muscle tissues in each group of mice (scale bar = 50 *μ*m); (b) pathological score in each group of mice was quantified; (c) W/D ratio of skeletal muscle was calculated to assess the extent of edema in each group of mice. The experiments were repeated three times. ^*∗*^*p* < 0.05, ^*∗∗*^*p* < 0.01.

**Figure 2:** (a, b, c, d) ELISA was conducted to determine the levels of inflammatory cytokines in the homogenate of mouse muscle tissues; (e) level of CK-MB was measured in the homogenate of mouse muscle tissues; (f) level of LDH was measured in the homogenate of mouse muscle tissues. The experiments were repeated three times. ^*∗*^*p* < 0.05, ^*∗∗*^*p* < 0.01.

**Figure 3:** (a) Immunofluorescent staining labeled pyroptosis marker caspase-1 was conducted to assess the extent of pyroptosis in each group of mice (scale bar = 50 *μ*m); (b) Western blot was used to examine the expression of pyroptosis markers in the muscle homogenate of each group of mice. The experiments were repeated three times. ^*∗*^*p* < 0.05, ^*∗∗*^*p* < 0.01.

**Figure 4:** (a) Immunofluorescent staining labeled autophagic markers Beclin-1 and LC3 was conducted to assess the extent of autophagy in each group of mice (scale bar = 50 *μ*m); (b) Western blot was used to examine the expression of autophagy markers in the mouse muscle homogenate. The experiments were repeated three times. ^*∗*^*p* < 0.05, ^*∗∗*^*p* < 0.01.

**Figure 5:** (a): Level of SOD was measured in muscle homogenate of each group of mice; (b) production of MDA was measured in muscle homogenate of each group of mice. The experiments were repeated three times. ^*∗*^*p* < 0.05, ^*∗∗*^*p* < 0.01.

**Figure 6:** (a, b) Western blot was used to examine the expression of HO-1, Nrf2, and NQO1 in the mouse muscle homogenate. The experiments were repeated three times. ^*∗*^*p* < 0.05, ^*∗∗*^*p* < 0.01.

## Data Availability

All data generated or analyzed during this study are available from the corresponding author upon reasonable request.
